# LH Pretreatment as a Novel Strategy for Poor Responders

**DOI:** 10.1155/2014/926172

**Published:** 2014-08-12

**Authors:** Anna Pia Ferraretti, Luca Gianaroli, Tatiana Motrenko, Elisabetta Feliciani, Carla Tabanelli, Maria Cristina Magli

**Affiliations:** ^1^SISMER, Reproductive Medicine Unit, Via Mazzini 12, 40138 Bologna, Italy; ^2^Human Reproduction Center, Prvomajska Street 4, 85310 Budva, Montenegro

## Abstract

*Introduction*. Poor response to ovarian stimulation is still a major problem in IVF. The study presents a new stimulation protocol evaluated in a suppopulation of very difficult young poor ovarian responders. *Material and Methods*. The study consists in two sections. The first includes data from a randomized controlled study involving forty-three young patients with a poor ovarian response in at least two previous cycles (intended as cycle cancellation or with ≤3 collected oocytes). Patients were randomized in two groups: group A (control) received FSH (400 IU/day), while group B received the new stimulation protocol consisting in a sequential association of 150 IU r-LH for 4 days followed by 400 IU r-FSH/after downregulation with daily GnRh agonist. The second includes data from the overall results in 65 patients treated with the new protocol compared to their previous performance with conventional cycles (historical control). *Results*. Both in the RCT and in the historical control study, LH pretreatment was able to decrease the cancellation rate, to improve the *in vitro* performance, and to significantly increase the live birth rates. *Conclusions*. LH pretreatment improved oocyte quantity and quality in young repeated poor responders selected in accordance with the Bologna criteria.

## 1. Introduction

Poor response to controlled ovarian hyperstimulation (COH) is one of the most challenging problems in assisted reproductive technology (ART). A variety of regimens have been proposed to improve poor responders' outcome, but results are often disappointing and controversial [1–5]. True poor ovarian responders (PORs) tend to react in a similar way under all conditions and protocols. This is not surprising if we consider that a poor response is the first clinical sign of a “not yet clinically evident” ovarian failure in which a reduced oocyte cohort cannot be reversed. In addition to a quantitative reduction of their oocyte cohorts, PORs present a high risk of implantation failure that may suggest a compromised oocyte quality [6]. Whereas in old women a poor oocyte quality is expected due to the biological ovarian aging, the oocyte quality still needs to be elucidated in young poor responders.

Egg donation is often offered as the only alternative to achieve positive results, but different stimulation protocols should be tested on young poor responders before abandoning the possibility of conceiving with their own gametes. Theoretically, if from poor responders patients it were possible to collect noncompromised and still competent oocytes that could produce good embryos for transfer, even though not numerous, an acceptable probability of pregnancy would exist for this category of patients. The optimal stimulation protocol has not been described yet, but it should be focused on the improvement of oocyte quality rather than quantity at collection.

For many years, the lack of a uniform definition of poor response was the most relevant factor that made it impossible to compare studies and very difficult to develop or assess any protocol to improve the outcome [1–5]. Recently, a consensus on the definition of PORs (the Bologna criteria) [7] was published as the first realistic attempt by a scientific community (ESHRE) to standardize the definition of POR. The aim was to identify women with a reduced ovarian reserve in a simple and reproducible manner for research purposes: to include homogeneous populations of women in future trials testing new strategies.

In the present study, a new protocol was tested in young PORs selected following at least two episodes of poor ovarian response after maximal stimulations. At the time of starting the study, the ESHRE PORs definition [7] was not yet available, but the methodology used for patients selection fulfilled the Bologna criteria since the beginning. The protocol consists of luteinizing hormone (LH) pretreatment on the rationale to use androgen-modulating agents to increase androgen accumulation in the micromilieu of preantral and small antral follicles.

The study was designed as a randomized controlled trial but, after the results analyzed in the first 43 patients, it was decided to stop the randomized study for ethical reasons and to use the new protocol in all the PORs.

Two sets of data will be therefore presented: the results of the randomized controlled trial (RCT) and the overall results in PORs undergoing the new protocol.

## 2. Material and Methods 

### 2.1. Randomized Controlled Trial

The study was performed between 2008 and 2010 at S.I.S.Me.R. (Società Italiana Studi di Medicina della Riproduzione), a private IVF centre in Italy. A total of 43 women aged ≤38 years with a history of repeated poor responses were selected for the study. All women had normoovulatory cycles, both ovaries, normal uterine cavity, and normal karyotype.

Indication for ART was a tubal factor in 21 cases, a male factor in 12, and tubal plus male factor in 10.

Before entering the study, each patient experienced at least two previous cycles with agonist or antagonist protocols and maximal FSH/HMG stimulation. All together, the patients experienced a total of 109 previous cycles where the cancellation rate was 51% (56/109) and the mean number of collected eggs was 2.5 ± 1 (range 0–3). Out of 40 embryo transfers (1.7 embryo/ET), three clinical pregnancies were obtained but all ended in early miscarriages.

At the time of planning the new attempt, patients were informed about the study and all accepted to be enrolled. Patients were then randomized in two treatment groups:

group A—control group (*n* = 21): maximal stimulation with 400 IU of rFSH per day (control group) in agonist downregulation (17 cycles) or antagonist protocol (4 cycles);

group B—study group (*n* = 22): pretreatment with rLH (150 IU/day for 4 days) preceding the administration of 400 IU/day of rFSH in agonist downregulation protocol.

Cycles were cancelled in the presence of <2 developing follicles; otherwise, 10.000 IU of HCG was administered when the leading follicle reached 18 mm in diameter. Egg retrieval was performed 36 hours later, and insemination was made by conventional IVF or ICSI depending on semen parameters.

Fertilization was assessed at approximately 16 hours after insemination, and embryos were evaluated at 24-hour time intervals by recording cell number and blastomere appearance and were consequently graded as I–IV (best–worst). Developing embryos were transferred on day 3, and the luteal phase was supported with 50 mg/day of progesterone in oil.

Except for the stimulation protocol, no different procedures were utilized in the two groups.

Before entering the study, all patients were tested for the ovarian reserve. During the study period, the only marker used was basal FSH. In all patients, blood levels of testosterone and DHEA were measured before starting the administration of rFSH.

Primary end points were considered the incidence of cycle cancellation and the live birth rate (LBR) per started cycle. Secondary end points included the number of collected eggs, the cleavage rate, and the implantation rate.

The study was approved by the local ethical committee.

Data were analysed by Student's *t*-test and *χ* ^2^ analyses as appropriate. Results are expressed as mean ± SD.

### 2.2. Overall Data with Historical Control

Between 2008 and 2012, the new protocol was utilized in a total of 79 cycles in 65 PORs (including the 22 patients from the RCT trial) aged ≤38 years and all selected after at least two previous poor ovarian responses (according to the Bologna criteria). Before entering the study, the patients experienced a total of 154 previous cycles performed using different stimulation protocols, including agonist and antagonist protocols with maximal stimulation as well as mild to minimal stimulations. No term pregnancies were obtained. From 2011, AFC and/or AMH were also utilized in addition to basal FSH to test the ovarian reserve.

## 3. Results 

### 3.1. Randomized Controlled Trial

Patients' age did not differ between the two groups as well as the infertility factor's distribution. The mean basal levels of FSH were 13.2 ± 7 mIU/mL in group A and 14.7 ± 10 mIU/mL in group B but, in total, 58% of these repeated PORs presented FSH levels > 12 mUI/mL.

The ovarian response is compared in Table 1. In group A, more cycles were cancelled compared to group B (43% versus 23%), but the difference was not statistically significant. In most of the egg retrievals (19/29), the numbers of eggs collected still remained in the range of poor response (≤3 oocytes) but a higher number of oocytes were collected in group B compared to group A (3.5 ± 1.5 versus 2.4 ± 1, *P* < 0.05). The percentage of metaphase II oocytes did not show any difference between the groups. The levels of circulating androgens at the start of FSH stimulation did not differ between the two groups.

Data comparing the fertilization and cleavage rates, as well as the clinical outcome, are presented in Table 2.

The fertilization rate was similar in the groups, but a higher percentage of 2 PN oocytes showed subsequent cleavage in group B compared to group A, leading to a higher number of cycles to be transferred in the LH group (77% versus 48%, *P* < 0.05). The morphology of the transferred embryos looked very similar in the two groups, but their potential to implant seemed to be improved by the LH priming (28% versus 6%, *P* = 0.06). The live birth rate per patient was significantly higher in group B compared with group A (32% versus 5%, *P* < 0.05).

As shown in Table 3, no differences were found in group B between patients with normal and elevated basal value of FSH, with the only exception of the number of collected oocytes.

### 3.2. Overall Data

Cumulative results obtained in the 65 PORs patients using the LH pretreatment are presented in Table 4 and compared with the results in their previous 154 cycles as historical control.

Out of the new patients entering the study from 2011 and tested with AMH or AFC, 86% presented abnormal results (AMH < 1 ng/mL or AFC < 7), confirming that these new markers are more accurate than basal FSH in evaluating the true ovarian reserve [8].

Compared to their historical control, the new regimen was able to decrease significantly the cancellation rate (*P* < 0.001) and to increase significantly the number of retrieved oocytes (*P* < 0.05) and the implantation rate (*P* < 0.001). The performance observed in this larger group of patients reproduced the preliminary results observed in the RCT, confirming that LH priming produced higher probability to conceive in these very difficult young PORs.

## 4. Discussion

Several strategies have been proposed for the management of poor responders, but results are often controversial [1–5]. For many years, the most important reason for that was the lack of a uniform and universally accepted definition of poor response, making many clinical trials not comparable because of the different inclusion criteria of the studied population.

In the present study, the studied population represents a homogeneous group of women with a premature reduction of the ovarian reserve selected according to the Bologna criteria [7]. With regard to pregnancy prospects, it is well known that PORs have poorer prognosis compared to normal responders [9], but they are not homogeneous groups of women. Among the factors predicting the final outcome, female age plays a crucial role. In their first cycle, young (<36 yrs) PORs have a pregnancy rate ranging from 5 to 35% [9]. But the present study, including only PORs who failed to conceive after at least two previous cycles, is dealing with a particularly difficult population of young PORs. Finally, the new stimulation protocol was first tested in a randomized controlled study and not only in comparison with the previous patients' performance (historical control). Possible bias and criticism related to patients' selection and study design were therefore prevented and the results can strongly support the hypothesis that LH pretreatment is able to improve oocyte number and oocyte quality in young repeated PORs, leading to favourable live birth rates.

Limitation of present study still remains small number of subjects caused by strict criteria used to select patients. However, most of the randomized controlled trials published to test new strategies in PORs and used to perform systematic reviews are including similar number of patients who were also selected using variable definition of PORs [5, 10]. Performing large-scale RCTs appears very difficult when dealing with this special category of patients who failed several previous cycles because of reduced ovarian reserve.

When the study was designed in 2008, very few studies were available in the literature based on the concept to test the androgen priming in PORs. Up to date, the use of androgen (testosterone, DHEA) or androgen modulating agents (aromatase inhibitors, LH, and HCG) represents one of the most interesting areas under investigation on the management of PORs. However, a recent review on the topic concluded that the evidence available is still limited and controversial [10].

The scientific background for this approach is quite extensive. Androgens receptors are abundant in the granulosa cells (GC) of healthy preantral and antral follicles of rhesus monkeys and their expression is upregulated by androgen administration [11, 12]. Accumulation of androgens in the micromilieu of the primate ovary plays a crucial role in early follicular development and GC proliferation [13]. Androgens excess stimulates early stage of follicular growth and increases the number of preantral and antral follicles [14, 15]. Increased intraovarian concentration of androgens augments FSH receptor expression in GC and, thus, potentially leads to enhanced responsiveness of ovaries to FSH [12]. In murine model, a positive correlation was found between androgen receptor and FSH receptor expression [16]. Similar findings were observed in humans [17]. In summary, prior to serving as a substrate for E2 synthesis in larger follicles, androgens may have a specific antiapoptotic action in preantral and small antral follicles.

Based on these considerations, poor responders represent the ideal patients to explore the concept of increasing the number of recruitable follicles after androgen priming. One of the potential effects under evaluation is the ability of androgens priming to increase the number of recruitable follicles by subsequent FSH stimulation. Studies using transdermal testosterone administration before ovarian stimulation are testing this concept with the aim to increase the number of follicles developing from very early stage (primary or even primordial??) to the stage sensitive to FSH/LH. To reach such effect, the priming should obviously last several weeks. A second potential effect to test is the effect of androgen priming in later stage of developing follicles: small antral follicles or secondary preantral follicles. To test this concept, even a short LH priming on follicles already sensitive to gonadotropins can be sufficient to induce a moderate (excessive can be detrimental!) increase of the level of androgens in their micromilieu.

In the present clinical study, the short LH pretreatment was able to reduce the cancellation rate and to increase the number of collected oocytes compared to controls, but actually most of the patients still remained in the range of a poor response (≤3 eggs). The new strategy did not show an evident positive effect in terms of “quantity.” The most relevant finding observed was the ability of LH pretreatment to improve the “oocyte quality,” as demonstrated by increased* in vitro *embryo development and implantation rate in group B compared to group A in the RCT and compared to previous cycles in the overall results. These very difficult young PORs were finally exposed to a probability to conceive similar to normal responders, despite their reduced ovarian reserve.

Poor responders are patients with aging ovaries, and LH receptors have been demonstrated to diminish with age [18, 19]. Based on this concept, addition of LH during FSH stimulation has been tested in PORs [20] but no beneficial effect on embryo quality was observed. The originality of the present study consists in the administration of LH “before” (and not “during”) FSH stimulation, with the aim to potentiate the intraovarian LH/androgen system in preantral and small antral follicles. However, only some hypothesis can be postulated to explain the positive action on oocyte quality and embryo viability in PORs. The whole maturation process of human oocytes is very complex and not yet understood. During the growth period, the oocyte increases in volume and synthesizes and accumulates products that are fundamental for its future, and cytoplasmic organelles undergo replication. Only mature, competent oocytes can resume meiotic maturation, complete the first mitotic cell cycles, and initiate the processes that bring to further development, including modifying chromatin structure and epigenetic status, activating the embryonic genome, and initiating the transcription of the array of genes that control the beginning of the developmental programme. According to some experimental data [21–25], COH may interfere with these delicate processes in the last phase of the oocyte growth. Most women undergoing ART are able to establish a new equilibrium following the interferences caused by COH and to produce competent oocytes and viable embryos. However, patients with already compromised ovaries might face up to difficulties in adapting to the new environment.

It could be speculated that some poor responders not only have a reduced cohort of follicles to be recruited by FSH, but also present some borderline maturation defect at the early stages of oocyte development that could alter the imprinting and/or gene expression mechanisms. These defects, if not corrected when still reversible, could be amplified by the hormonal environment induced by FSH stimulation, leading to a drastic reduction in the generation of viable embryos. Exposure of small follicles to LH prior to FSH recruitment seems to adjust this process by improving the oocyte cytoplasmic maturation and, therefore, the future embryogenesis. In agreement with these considerations, it was reported in a previous study that supplementing* in vitro*-maturation medium with high concentrations of LH added to FSH improved embryonic development of IVM human and bovine oocytes [26].

Some authors [27] are proposing to use mild stimulations in PORs on the principle to avoid adding exogenous FSH while endogenous FSH is already elevated. This strategy has to be tested in prospective controlled studies on homogeneous populations of PORs to evaluate if and which subcategories of PORs could have better prognosis of pregnancy with this protocol. Actually, most of the patients included in our study experienced already mild/minimal stimulations in the several cycles performed before entering the new LH pretreatment protocol, without any success. Some very difficult PORs may need maximum stimulation to develop even few follicles, but excessive FSH stimulation can negatively affect oocyte quality [28]. On this scenario, we decided to test the LH pretreatment before maximum FSH stimulation and the results seem to suggest a protective role against the negative effect of the high FSH doses required.

The similar blood levels of androgens observed in groups A and B of the RCT were not surprising: LH priming on the micromilieu of preantral and small antral follicles cannot increase the circulating androgen levels.

There was a doubt is positive effect produced by LH priming or FSH receptors desensitizing caused by GnRH agonist down regulation in trial group. Having in mind that those patients had previously at least two IVF attempts with protocol including agonist downregulation, as well as the fact that for 81% of patients in group A (control group) long protocol was used, difference in oocyte quality and increased pregnancy rate should be addressed to LH priming.

Finally, when comparing patients with elevated or normal basal FSH level, the results observed are in agreement with previous reports, suggesting that the elevation of FSH in cycling women may be more related to a quantitative rather than a qualitative decline of the ovarian reserve [29]. In other words, elevated levels of basal FSH in young and repeated poor responders should not be considered as* a priori* disqualifying reason from further IVF attempts [28, 30]. The same has to be true for the new ovarian reserve tests (AMH and AFC), more sensitive than FSH in predicting the ovarian response, but not accurate markers of oocyte quality and pregnancy prognosis.

In summary, the diminished follicle cohort in poor responders cannot be significantly overcome by the use of LH/androgen priming strategies, but, in very difficult young PORs who experienced repeated cycles with different protocols (from maximum to mild stimulation) without conception, LH pretreatment can improve oocyte quality or reverse some borderline defects than can be induced by maximal FSH stimulation. Since oocyte “age” is still acceptable, the “correction” of such defects can allow good prognosis of pregnancy, despite the low number of eggs.

Further investigation on the efficacy of LH pretreatment is needed, although larger clinical trials could not be sufficient to definitively address the several questions that are still open on ovarian stimulation. Only studies taking into consideration the molecular basis of the hormone action (gene expression, methylation status, and proteomics) will be able to clarify the clinical results obtained in the controversial area of poor responders.

## 5. Conclusions

In this study, we showed that LH pretreatment, in repeated poor responders, produced a small increase in the number of oocytes retrieved but a relevant improvement of their quality. Young poor responders may thus benefit from the use of this new stimulation protocol, although further studies are needed to support these clinical results.

## Figures and Tables

**Table 1:** Results of the randomized controlled trial: ovarian response.

	Group A	Group B	*P* value
Number of patients	21	22	
Age	34.8 ± 3.6	34.3 ± 3.7	n.s.
Number of cancelled cycles (%)	9 (43%)	5 (23%)	n.s
Total IU of rFSH	3906 ± 1367	4152 ± 1429	n.s
Estradiol on HCG day (pg/mL)	651 ± 150	725 ± 150	n.s.
Number of collected oocytes	31 (2.4 ± 1)	58 (3.5 ± 1.7)	<0.05
Number of metaphase II oocytes (%)	27 (87%)	52 (89%)	n.s
Testosterone (ng/mL) at the start of FSH stimulation	0.43 ± 0.23	0.39 ± 0.18	n.s
DHEA (ng/mL) at the start of FSH stimulation	7.2 ± 2.66	7.5 ± 3.54	n.s

**Table 2:** Results of the randomized controlled trial: *in vitro* performance and final outcome.

	Group A	Group B	*P* value
Number of eggs retrievals	12	17	
Fertilization rate	86 (24/28)	90 (47/52)	n.s
Cleavage rate	71 (17/24)	91 (43/47)	<0.05
% of grade 1 embryos	70 (12/17)	81 (35/43)	n.s
Number of transferred cycles (% on started cycles)	10 (48%)	17 (77%)	<0.05
Number of transferred embryos (mean embryos/transfer)	16 (1.6)	35 (2.0)	
Number of clinical pregnancies	1	8	
Implantation rate	6 (1/16)	29 (10/35)	0.06
Number of early miscarriages	0	1	
Live birth rate/patient (%)	5 (1/21)	32 (7/22)	0.025

**Table 3:** Results in the LH pretreatment group according to basal FSH value.

	FSH ≥ 12 mUI/mL	FSH < 12 mUI/mL
Number of patients (age)	9 (35.7 yrs)	13 (35.5 yrs)
Number of retrievals	7	10
Mean number of recovered eggs	2.5 ± 1.0	3.8 ± 1.2
Number of transferred cycles	7	10
Number of clinical pregnancies	3	5
Implantation rate (%)	27 (3/11)	29 (7/24)
Live birth rate/patient (%)	30 (3/9)	31 (4/13)

**Table 4:** Overall results in the 65 PORs.

	LH pretreatment	Previous cycles
Cycles	79	154
Cancellation rate	22% (17)	51% (79)
Number of collected oocytes	3.5 ± 1.9	2.5 ± 1.2
Fertilization rate	80% (141/176)	83% (135/163)
Cleavage rate	92% (130/141)	62% (84/135)
Transferred cycles (mean embryos/ET)	54 (1.7 ± 0.5)	58 (1.5 ± 0.5)
Implantation rate	22.3% (23/103)	4% (4/89)
Clinical pregnancy rate/ET	37% (20/54)	7% (4/58)
Early miscarriages	1	4
Live birth rate/started cycle	24%	0%
Live birth rate/patient	29%	0%
